The article "Association of Platelet-to-Lymphocyte Ratio with Stroke-Associated Pneumonia in Acute Ischemic Stroke" was published in 2022. Journal: J Healthc Eng.

# Association of Platelet-to-Lymphocyte Ratio with Stroke-Associated Pneumonia in Acute Ischemic Stroke

**DOI:** 10.1155/2022/1033332

**Published:** 2022-03-18

**Authors:** Wei Li, Cailian He

**Affiliations:** Department of Neurology, Beijing Shijitan Hospital, Capital Medical University, Beijing 100038, China

## Abstract

A common consequence of acute ischemic stroke (AIS), stroke-associated pneumonia (SAP), might result in a poor prognosis after stroke. Based on the critical position of inflammation in SAP, this study aimed to explore the correlation between platelet-to-lymphocyte ratio (PLR) and the occurrence of SAP. We included 295 patients with acute ischemic stroke, 40 with SAP, and 255 without SAP. The area under the receiver operating characteristic curve was used to determine the diagnostic value of SAP risk factors using binary logistic regression analysis. The comparison between the two groups showed that age, the baseline National Institutes of Health Stroke Scale (NIHSS) score, and the proportion of dysphagia, atrial fibrillation, and total anterior circulation infarct were higher, and the proportion of lacunar circulation infarct was lower in the SAP group (*P* < 0.001). In terms of laboratory data, the SAP group had considerably greater neutrophil counts and PLR, while the non-SAP group (*P* < 0.001) had significantly lower lymphocyte counts and triglycerides. Binary logistic regression analysis revealed that older age (aOR = 1.062, 95% CI: 1.023–1.102, *P* = 0.002), atrial fibrillation (aOR = 3.585, 95% CI: 1.605–8.007, *P* = 0.019), and PLR (aOR = 1.003, 95% CI: 1.001–1.006, *P* = 0.020) were independent risk factors associated with SAP after adjusting for potential confounders. The sensitivity and specificity of PLR with a cutoff value of 152.22 (AUC: 0.663, 95% CI: 0.606–0.717, *P* = 0.0006) were 57.5% and 70.6%, respectively. This study showed that high PLR is an associated factor for SAP in AIS patients. Increased systemic inflammation is linked to SAP in ischemic stroke. Inflammatory biomarkers that are easily accessible may aid in the diagnosis of high-risk SAP patients.

## 1. Introduction

Stroke is a common and leading cause of death and disability worldwide, imposing a heavy burden on society and the economy [1, 2]. Stroke-associated pneumonia (SAP) often occurs after a stroke; approximately 7%–38% [3–8] of stroke patients are diagnosed with SAP during hospitalization. Once a patient develops SAP, it leads to a poor prognosis and a prolonged hospital duration [9–12].Early diagnosis and preventive treatment are necessary for patients at high risk of SAP. Therefore, an effective biomarker is needed for risk assessment and early detection of SAP. Neurogenic immunosuppression is one of the critical mechanisms of increased susceptibility to postinfection [13, 14].

The article "Association of Platelet-to-Lymphocyte Ratio with Stroke-Associated Pneumonia in Acute Ischemic Stroke" was published in 2022. Journal: J Healthc Eng.

Platelet-to-lymphocyte ratio (PLR) is a novel and inexpensive biomarker that reflects systemic inflammation response [15, 16], which is affected by changes in lymphocytes and platelets after acute stroke. PLR is a sensitive marker to predict the occurrence and prognosis of cardiovascular events [16, 17], cerebrovascular diseases [18], poststroke depression [19],and pneumonia [20]. However, the association of PLR with SAP is uncertain. In light of this, we investigated the relationship of PLR with SAP in AIS patients.

In the proposed investigation, we discovered that high PLR is linked to SAP in AIS patients. PLR could be a useful tool for identifying high-risk SAP patients. It is more beneficial to improve results if SAP is detected early and well prevented. PLR was found to be considerably greater in the SAP group than in the non-SAP group in this study.

In the following section, we discuss the section-wise study.  Section 2 discusses the materials and methods and also discusses the study subjects, clinical variables collection, laboratory parameters and clinical features, statistical analysis, and results.  Section 3 defines the conclusion of the study. Finally, the research work is concluded in Section 4.

## 2. Materials and Methods

The overall quality of any research dissemination output is evaluated in this section and it reveals to readers what techniques, methodologies, designs, and treatments are used in the research, allowing us to repeat the results.

### 2.1. Study Subjects

Acute ischemic stroke patients in the Department of Neurology, Beijing Shijitan Hospital, were included in this study between March 1, 2018, and July 31, 2019. The study protocol was approved by the Scientific Research Ethics Committee of Beijing Shijitan Hospital Affiliated with Capital Medical University.

The inclusion criteria for enrolled patients are as follows:

1. Hospitalization within 72 h after the onset of symptoms
2. Patients diagnosed as new acute ischemic stroke by imaging examination (cranial magnetic resonance imaging or computed tomography) at the time of admission
3. Modified Rankin scale (mRS) score<2 before admission
4. Patients who were not discharged within 3 days before hospitalization

The exclusion criteria are as follows:

1. The acute infections (vacuities, urinary, and infection of the upper or lower respiratory tract) within 2 weeks before the onset of the stroke
2. Medical history of cancer, hematologic disease, severe liver and kidney dysfunction, and autoimmune disease

### 2.2. Clinical Variables Collection

Demographic data obtained at admission include age, sex, and the length of hospitalization. Premorbid history relevant risk factors contain current smoking, coronary heart disease, hypertension, diabetes, previous stroke, and atrial fibrillation.

The article "Association of Platelet-to-Lymphocyte Ratio with Stroke-Associated Pneumonia in Acute Ischemic Stroke" was published in 2022. Journal: J Healthc Eng.

### 2.3. Laboratory Parameters and Clinical Features

Within 24 h after admission, peripheral venous blood was collected from the participants and used for immediate biomarker detection. Laboratory data consisted of neutrophils, lymphocytes, platelets, total cholesterol (TC), triglycerides (TG), and low-density lipoprotein cholesterol (LDL-C). The PLR (defined as platelet/lymphocyte) was calculated. The clinical features of patients included dysphagia, the Oxfordshire Community Stroke Project (OCSP), and baseline National Institutes of Health Stroke Scale (NIHSS) score on admission.

According to clinical and laboratory examinations and chest X-ray or CT scan results retrospectively gathered from medical records, SAP was defined as a lower respiratory tract infection within the first 7 days of hospitalization after a stroke [21, 22].

### 2.4. Statistical Analysis

Normally distributed continuous variables were expressed as the mean ± standard deviation, while nonnormally distributed variables were expressed as the median (interquartile range). The Mann–Whitney *U* test was used to compare the clinical characteristics of continuous variables between groups. The chi-square test was used for categorical variables. Variables with *P* < 0.05 from the results of the univariate analyses were considered confounders in the multivariable logistic regression analysis. The association between different PLR and SAP risks was estimated using univariate analysis and binary logistic regression analysis. All patients were classified into two groups according to their median PLR (126.67), and the potential confounders of PLR were identified. We adjusted all potential confounding factors (parameters with *P* < 0.05 in univariate analysis). The results are presented in the form of an adjusted odds ratio (aOR) and 95% confidence interval (CI).

We conducted the receiver operative curve (ROC) and the area under the curve (AUC) to measure the specificity and sensitivity of PLR and obtained the optimal cutoff value of PLR. Results were considered significant at *P* < 0.05. The analysis of ROC was performed with MedCalc 15.6 (MedCalc Software, Belgium). Other statistical analyses were carried out using SPSS v23 (SPSS Inc., Chicago, IL).

## 3. Results

A total of 295 consecutive AIS patients were retrospectively included from March 1, 2018, and July 31, 2019, according to the inclusion and exclusion criteria, 40 (13.6%) of whom were diagnosed with SAP in the final analysis (Figure 1). The average age of patients was 69.5 ± 12.0 years, and 196 (66.4%) were male. The median length of hospitalization was 14.0 (11.0, 17.0) days. The comparison of demographic, clinical, and laboratory characteristics is given in Table 1. There were significant differences in age (*P* < 0.001) and baseline NIHSS score (*P* < 0.001) between the SAP group and the non-SAP group. The presence of dysphagia (*P* < 0.001), atrial fibrillation (*P* < 0.001), total anterior circulation infarction (TACI) (*P* < 0.001), and lacunar circulation infarction (LACI) (*P* < 0.001) were significantly different between the two groups. Neutrophil counts and PLR were significantly increased (*P* ≤ 0.001; Figure 2), whereas lymphocyte counts and TG were significantly decreased in the SAP group (*P* < 0.001). The number of platelets in the patients with SAP was decreased, although not statistically significant.

The article "Association of Platelet-to-Lymphocyte Ratio with Stroke-Associated Pneumonia in Acute Ischemic Stroke" was published in 2022. Journal: J Healthc Eng.

The demographic and clinical characteristics (parameters with *P* < 0.05 in univariate analysis) in the high and low PLR groups are given in Table 2. We found that patients with the high PLR had high baseline NIHSS scores (*P* = 0.047) and low TG (*P* = 0.004). The prevalence of dysphagia (*P* = 0.020) was significantly higher in the high PLR group than in the low PLR group.

In the univariate analysis, the variables with *P* < 0.05 were used as covariates, and SAP was used as a dependent variable. As given in Table 3, after adjusting for the confounders of PLR, multivariate logistic regression analysis showed that PLR (aOR = 1.003, 95% CI: 1.001–1.006, *P* = 0.020), age (aOR = 1.062, 95% CI: 1.023–1.102, *P* = 0.002), and atrial fibrillation (aOR = 3.585, 95% CI: 1.605–8.007, *P* = 0.019) remained associated with SAP. In the ROC analysis, the best cutoff level of PLR was 152.22 (*P* = 0.0006), with 0.575 sensitivity and 0.706 specificity. The area under the ROC curve was 0.663 (95% CI: 0.606–0.717) (Figure 3).

## 4. Discussion

Based on increasing evidence, researchers reported the predictive effectiveness of PLR in the prognosis of artery diseases [16–18] and inflammation diseases. With reference to the studies by Turkmen et al. and Uslu et al. [23, 24] in the present study, we found that high PLR is associated with SAP in AIS patients. The results of multivariate analysis showed that PLR, a marker of systemic inflammation, is an independent risk factor for SAP, which further confirmed high PLR may be used as an effective indicator of inflammatory diseases.

Platelets have the function of regulating inflammation and immune responses, which play an important role in the formation of thrombosis in the arterial circulation. When AIS occurs, abnormal platelets are overactivated and accumulated [25], which may lead to thrombosis and vascular blockage and then vascular events [26]. Changes in circulating platelet counts are uncertain in diverse diseases. Platelets can increase in many inflammations with an acute phase. In the case of sepsis, the platelet count will increase due to the accelerated expression of platelets after the increase in their breakdown [27]. However, we found the platelet counts were decreased in AIS patients with SAP. There could be three reasons for this observation. The first reason is the particularities of AIS patients. When arterial platelet-fibrin thrombi are formed in AIS patients, a reduction of the circulation platelet counts occurs due to their increased consumption in the infarction area [28]. The second reason is that platelet count in AIS patients may correlate with disease severity. Ming Yang et al. showed that AIS patients in the lowest platelet count quintile had a higher risk of poor functional outcome [29]. In this study, SAP patients were severe, with high admission NIHSS scores, which lead to the reduction of platelet count. The third reason may be the effect of antithrombotic therapy of acute AIS on platelets. IVT using rt-PA influences peripheral blood platelet counts and lymphocyte concentrations, resulting in enhancing infection risk [30].

The article "Association of Platelet-to-Lymphocyte Ratio with Stroke-Associated Pneumonia in Acute Ischemic Stroke" was published in 2022. Journal: J Healthc Eng.

The lymphocytes belong to the adaptive immune cells, which influence the regulation of the inflammatory response. Lymphocytes were suggested to be a pivotal subtype that determined the severity of neuroinflammation in acute brain injuries. Urra et al. [31] suggested that lymphopenia in the early stages of stroke is a sign of persistent brain damage, stress response, and a greater possibility of infection. In addition, it has been reported that lymphopenia after reperfusion in vascular events can effectively predict the existence of microvascular occlusion in the early stage [32]. Konstantin et al. [33] reported apoptosis of lymphocytes after stroke, and catecholamine-mediated lymphocyte defect played an important role in stroke-associated infection. Recent studies in rodent models have shown that T cells accumulate early in the damaged area within the first 24 hours after the onset of a stroke, which causes lymphopenia in peripheral blood [34]. The stroke-induced lymphocyte apoptosis results in immune system suppression and inflammation [35, 36], shifting from a proinflammatory Th1 type response to an anti-inflammatory Th2 type response. Therefore, stroke causes local inflammation and leads to stroke-induced immunosuppressive syndrome (SIDS) [14]. SIDS then leads to the systemic inflammatory response through endocrine pathways involving the hypothalamic-pituitary-adrenal axis or activation of the sympathetic nervous system [33, 37, 38]. Meanwhile, SIDS results in decreased peripheral blood lymphocyte counts and functional T cell inactivation [39]. The results of this study further supported that lymphopenia caused by immunosuppression after stroke has a potential effect on SAP susceptibility.

The article "Association of Platelet-to-Lymphocyte Ratio with Stroke-Associated Pneumonia in Acute Ischemic Stroke" was published in 2022. Journal: J Healthc Eng.

PLR is a systemic inflammation index, which is calculated by dividing the platelet count by lymphocyte count. PLR represents the burden of systemic inflammation and combines platelet counts and lymphocytes counts to predict the prognosis of cardiovascular diseases [40] and ischemic stroke [41]. Altintas et al. found that high PLR values could reflect the infarcted size and poor recanalization rate in patients with thrombectomy therapy, supporting the view that PLR represents a prothrombotic inflammatory state [40]. In addition, PLR may provide important information for pulmonary diseases. Kumar et al. [42] showed that PLR could predict the 90-day mortality in patients with acute exacerbations of COPD. The PLR value can guide in diagnosing hypersensitivity pneumonia [43]. Kartal et al. showed that utilization of PLR may differentiate patients with community-acquired pneumonia [44]. Moreover, Jong-Han Lee et al. detected PLR might have diagnostic utilities such as CRP in the evaluation of the severity of pneumonia patients [45]. CRP has been reported to have a significant prognostic value and a useful adjunctive test as well as being a marker of treatment response in inflammation disease. The ability of PLR to predict infectious diseases is further proved by this indirect evidence. PLR was found to be considerably greater in the SAP group than in the non-SAP group in this study. However, Ahmet Adiguzel et al. found no correlation between the PLR level and SAP [46]. The possible reason for the different results is the difference in the severity of the stroke patients included. They included stroke patients with NIHSS >10 who were sicker than the patients in our study. Based on the discussion above, we speculated that there may be a correlation between high PLR and the occurrence of SAP, helping clinicians assess high-risk SAP in clinical works. The followings could be viewed as potential limitations to the study. First, selection bias is a concern because we undertook a single-center retrospective study. This study would have been more convincing if our sample size was enlarged. Second, as a retrospective study, some acute inflammation biomarkers were not incorporated for analysis. This could have a certain impact on the result. We will conduct prospective studies in the future to further prove this conclusion. Third, PLR was only measured at admission. Given the limitations related to the retrospective design, no data evaluating the dynamic change of PLR were available. In future studies, the hematologic markers during hospitalization should be dynamically measured to evaluate the predictive value of PLR for SAP. Fourth, we cannot rule out residual confounding or the effect of unmeasured confounders. Further studies need to record more potential risk factors for SAP.

The article "Association of Platelet-to-Lymphocyte Ratio with Stroke-Associated Pneumonia in Acute Ischemic Stroke" was published in 2022. Journal: J Healthc Eng.

## 5. Conclusion

In conclusion, our study showed that high PLR is associated with SAP in AIS patients. PLR may be a promising indicator to identify high-risk SAP patients. High PLR was found to be a risk factor for SAP in AIS patients in this investigation. In ischemic stroke, increased systemic inflammation is connected to SAP. Easy-to-find inflammatory biomarkers could aid in the diagnosis of high-risk SAP patients. It is more beneficial to improve results if SAP is detected early and well prevented.

## Figures and Tables

**Figure 1:** Flow diagram of the patient selection process.

**Figure 2:** PLR levels and SAP. Violin plot of PLR distribution in patients with SAP and without SAP.

**Figure 3:** The receiver operating characteristic (ROC) curve analysis of platelet-to-lymphocyte ratio for predicting SAP.

**Table 1:** Comparison of the characteristics of AIS patients according to the onset of SAP.

Characteristics	Total (*N* = 295)	Non-SAP (*N* = 255)	SAP (*N* = 40)	*P* value
Age, years, mean ± SD	69.5 ± 12.0	68.1 ± 11.7	77.5 ± 10.6	<0.001*∗*
Male, *n* (%)	196 (66.4)	171 (67.1)	25 (62.5)	0.570
Length of hospitalization, days, median (IQR)	14.0 (11.0, 17.0)	14.0 (11.0, 16.0)	14.5 (9.0, 33.0)	0.241
Baseline NIHSS, median (IQR)	3 (1, 7)	3 (1, 5)	14 (7, 18)	<0.001*∗*
Dysphagia, *n* (%)	49 (16.6)	15 (5.8)	34 (85.0)	<0.001*∗*
Current smoking, *n* (%)	96 (32.5)	85 (33.3)	11 (27.5)	0.464
Coronary artery disease, *n* (%)	88 (29.8)	72 (28.2)	16 (40.0)	0.131
Hypertension, *n* (%)	229 (77.6)	196 (76.9)	33 (82.5)	0.426
Diabetes, *n* (%)	106 (35.9)	96 (37.6)	10 (25.0)	0.121
Previous stroke, *n* (%)	81 (27.5)	66 (25.9)	15 (37.5)	0.126
Atrial fibrillation, *n* (%)	46 (15.6)	29 (11.4)	17 (42.5)	<0.001*∗*
OCSP				
TACI, *n* (%)	15 (5.1)	5 (2.0)	10 (25.0)	<0.001*∗*
PACI, *n* (%)	90 (30.5)	78 (30.6)	12 (30.0)	0.940
POCI, *n* (%)	39 (13.2)	30 (11.8)	9 (22.5)	0.062
LACI, *n* (%)	151 (51.2)	142 (55.7)	9 (22.5)	<0.001*∗*
TC, mmol/L, median (IQR)	4.2 (3.5, 5.0)	4.3 (3.6, 5.0)	4.0 (3.1, 4.9)	0.086
TG, mmol/L, median (IQR)	1.2 (0.9, 1.7)	1.3 (1.0, 1.8)	0.9 (0.7, 1.3)	<0.001*∗*
LDL-C, mmol/L, median (IQR)	2.4 (1.8, 3.0)	2.4 (1.8, 3.0)	2.2 (1.8, 2.8)	0.306
Neutrophils, ×10^9^/L, median (IQR)	4.3 (3.3, 6.0)	4.0 (3.1, 5.3)	7.3 (6.0, 9.6)	<0.001*∗*
Lymphocytes, ×10^9^/L, median (IQR)	1.6 (1.3, 2.1)	1.8 (1.4, 2.1)	1.1 (0.9, 1.6)	<0.001*∗*
PLT, ×10^9^/L, median (IQR)	216.0 (179.0, 253.0)	216.0 (180.0, 253.0)	210.5 (152.3, 247.8)	0.137
PLR, median (IQR)	126.7 (99.6, 175.3)	123.2 (98.0, 163.8)	161.2 (114.1, 209.2)	0.001*∗*

NIHSS, National Institute of Health Stroke Scale; OCSP, Oxfordshire Community Stroke Project; TACI, total anterior circulation infarct; PACI, partial anterior circulation infarct; POCI, posterior circulation infarct; LACI, lacunar circulation infarct; TC, total cholesterol; TG, triglycerides; LDL-C, low-density lipoprotein cholesterol; PLT, platelet; PLR, platelet-to-lymphocyte ratio; SD, standard deviation; IQR, interquartile range; SAP, stroke-associated pneumonia. *∗P* values less than 0.05 were considered statistically significant.

The article "Association of Platelet-to-Lymphocyte Ratio with Stroke-Associated Pneumonia in Acute Ischemic Stroke" was published in 2022. Journal: J Healthc Eng.

**Table 2:** Comparison of the characteristics between subgroups based on the median PLR.

Characteristics	Low PLR	High PLR	*P* value
	*N* = 147 (PLR<126.67)	*N* = 148 (PLR≥126.67)	
Age, years, mean ± SD	68.8 ± 12.2	70.0 ± 11.7	0.346
Baseline NIHSS, median (IQR)	3 (1, 5)	4 (2, 8)	0.047^*∗*^
Dysphagia	17 (11.6)	32 (21.6)	0.020^*∗*^
Atrial fibrillation, *n* (%)	17 (11.6)	29 (19.6)	0.057
TG, mmol/L, median (IQR)	1.2 (1.0, 1.8)	1.1 (0.8, 1.6)	0.004^*∗*^

NIHSS, National Institute of Health Stroke Scale; TG, triglycerides; PLR, platelet-to-lymphocyte ratio; SD, standard deviation; IQR, interquartile range. ^*∗*^*P* values less than 0.05 were considered statistically significant.

**Table 3:** Multivariate logistic regression analysis of the associations between PLR and SAP.

Risk factors	B	SE	Wald	*P* value	aOR	aOR (95% CI)
Age	0.060	0.019	9.819	0.002^*∗*^	1.062	1.023–1.102
Atrial fibrillation	1.277	0.410	9.699	0.019^*∗*^	3.585	1.605–8.007
PLR	0.003	0.002	5.393	0.020^*∗*^	1.003	1.001–1.006

PLR, platelet-to-lymphocyte ratio; SAP, stroke-associated pneumonia; SE, standard error; aOR, adjusted odds ratio. ^*∗*^*P* values less than 0.05 were considered statistically significant.

## Data Availability

The datasets used to support the findings of this study are available from the corresponding author upon request.
